This article has been retracted.

# Efficacy and Safety of Peptide Receptor Radionuclide Therapy for the Treatment of Pancreatic Neuroendocrine Tumors: A Systematic Review and Meta-Analysis of Comparative Studies

**DOI:** 10.7759/cureus.80817

**Published:** 2025-03-19

**Authors:** Jun Zhao, Xiaxia Pei, Yumin Li

**Affiliations:** 1 Department of General Surgery, Second Hospital of Lanzhou University, Lanzhou, CHN; 2 Department of Oncology, Second Hospital of Lanzhou University, Lanzhou, CHN; 3 Key Laboratory of the Digestive System Tumors of Gansu Province, Second Hospital of Lanzhou University, Lanzhou, CHN

**Keywords:** cancer, meta-analysis, pancreatic neuroendocrine tumors, peptide-receptor radionuclide therapy, systematic review

## Abstract

Peptide receptor radionuclide therapy (PRRT) showed promising potential in the management of patients with pancreatic neuroendocrine tumors (pNETs). However, there is still a lack of evidence on its relative efficacy and safety compared with other treatment options. This review aims to synthesize the existing evidence on the efficacy and safety of PRRT for pNETs compared to different treatments. An electronic search was conducted from inception to May 2024. Comparative studies, including randomized controlled trials (RCTs), cohort studies, and case-control studies, that focused on the use of PRRT for treating pNETs were included. Efficacy outcomes included disease control rate (DCR), complete response (CR), partial response (PR), stable disease (SD), progression-free survival (PFS), and overall survival (OS). Safety outcomes were grade 3-4 hematological and renal toxicity and adverse events (AEs). Nine studies met the inclusive criteria. Among them, only one (11.1%) study was an RCT. Meta-analysis between full and reduced dosages of 177Lu-DOTATATE for G1-G2 pNETs revealed no significant differences in DCR, CR, PR, SD, and PFS between the groups. However, the full dosage group showed superior efficacy in some outcomes (DCR, CR, and PR). When PRRT was compared to other treatments such as surgery, chemotherapy, and targeted agents, it was associated with longer PFS and OS. Additionally, PRRT combined with capecitabine and salvage PRRT also showed efficacy in advanced cases. Safety analysis indicated that PRRT is well-tolerated, with minimal severe toxicity reported. PRRT is a promising therapeutic option for patients with advanced pNETs, offering a balance of efficacy and safety compared to other available treatments based on the low quality of evidence. Full-dosage PRRT may provide better outcomes than reduced dosages, and salvage PRRT remains effective for progressive disease. However, further high-quality RCTs are needed to confirm these findings and optimize PRRT usage in pNETs.

## Introduction and background

Pancreatic neuroendocrine tumors (pNETs) are a diverse group of neoplasms that originate from the endocrine cells of the pancreas. Although pNETs represent only a small percentage of pancreatic tumors, their incidence has been rising rapidly in recent years [1]. Data from the Surveillance, Epidemiology, and End Results (SEER) registries between 2000 and 2016 showed that the annual incidence of pNETs increased from 0.27 to 1.00 per 100,000 population, with a median overall survival (OS) of 68 months [2]. The clinical presentations and prognoses of pNETs varied based on differentiation, grading, and other molecular markers [3].

Current clinical guidelines recommend several treatment options for pNETs, including surgical resection, chemotherapy, and targeted therapies such as Everolimus and Sunitinib and peptide receptor radionuclide therapy (PRRT) [4-8]. PRRT is primarily indicated for patients with well-differentiated (G1-G2) [4], metastatic pNETs exhibiting high somatostatin receptor expression (e.g., confirmed by 68Ga-DOTATATE positron emission tomography/computed tomography), as recommended by the European Neuroendocrine Tumor Society (ENETS) and National Comprehensive Cancer Network (NCCN) guidelines [4,6]. Surgical resection remains the first-line option for localized disease, while PRRT is reserved for advanced or inoperable cases or those refractory to other therapies such as somatostatin analogs (SSAs), chemotherapy, or targeted agents. Among these, PRRT has emerged as an innovative and promising treatment. PRRT involves the use of radiolabeled somatostatin analogs, such as 177Lu-DOTATATE and 90Y-DOTATOC, which selectively target somatostatin receptors expressed on tumor cells. In 2017, the NETTER-1 trial [9] showed that 177Lu-DOTATATE significantly improved median progression-free survival (PFS) in patients with well-differentiated, metastatic midgut NETs compared to high-dose octreotide. In subgroup analysis, 177Lu-DOTATATE showed comparable efficacy for pNETs [10]. Subsequently, PRRT was first approved for the treatment of pNETs in Europe in 2017 [11] and received the Food and Drug Administration (FDA) approval in the United States in 2018 [12].

While PRRT has been incorporated into clinical guidelines for advanced pNETs, comparative studies evaluating its efficacy and safety against other treatments (e.g., surgery, chemotherapy, targeted therapy) remain limited. While observational studies [13,14] have indicated the benefits of PRRT in terms of tumor control and symptom relief, there is still a need for comprehensive data to fully assess its performance. Moreover, comparative studies between PRRT and other recommended treatments are limited, leaving questions about the relative advantages and disadvantages of various therapeutic approaches. Therefore, this systematic review and meta-analysis aims to synthesize the existing evidence on the efficacy and safety of PRRT for pNETs compared to different treatments.

## Review

Methodology

This study was pre-registered on the Open Science Framework (OSF) (osf.io/4u7t9). We followed the Preferred Reporting Items for Systematic Reviews and Meta-Analyses (PRISMA) statement [15] for reporting.

Inclusion and exclusion criteria

We included studies that met all the following criteria: the population consisted of patients diagnosed with pNETs aged ≥18 years (for metastatic NETs, the primary origin had to be the pancreas); the intervention/exposure was PRRT (including both alpha-emitters and beta-emitters); the control group received either a placebo, no intervention, other treatments (including SSAs, surgical resection, targeted agents, or chemotherapy), or different PRRT treatment protocols. Eligible studies had to report at least one of the following outcomes: disease control rate (DCR), complete response (CR), partial response (PR), stable disease (SD), progressive disease (PD), PFS, OS, toxicity, or adverse events (AEs). We included randomized controlled trials (RCTs), cohort studies, and case-control studies. Given the limited availability of comparative studies on this topic, we also included abstracts with sufficient data.

Studies were excluded if the effect of PRRT could not be isolated from other interventions (e.g., PRRT plus SSAs vs. SSAs alone) and if patients with pNETs could not be distinguished from those with other types of NETs (e.g., gastroenteropancreatic neuroendocrine tumors [GEP-NETs]) if there were duplicate publications, or if the study was not published in English.

Search strategy

We conducted a comprehensive search of electronic databases, including MEDLINE via PubMed, Embase, Web of Science, and Cochrane Library from inception to June 12, 2024. The search strategy combined MeSH terms and free-text terms relevant to pNETs and PRRT. Google Scholar, ClinicalTrials.gov, and the list of included references were also searched for supplementary data. The detailed search strategies for each database are provided in the Appendix.

Screening process

Two reviewers (Z, J, and P, X) screened titles and abstracts, followed by full texts independently according to the inclusion criteria. Discrepancies were resolved through consultation with a senior researcher (L, Y). A pilot selection with 100 records before the full screening was conducted before full screening to improve the consistency between the reviewers.

Data extraction

Two independent reviewers (Z, J and P, X) used a pre-defined extraction form (Microsoft Excel) to collect the following items: (1) study characteristics (first author, title, journal, publication year, study design, and conducted country); (2) patients characteristics (detailed type of pNETs, sample size, age, and gender); (3) interventions/exposures and controls (treatment protocols, including dosage, cycles, and follow-up duration); (4) outcomes at the end of treatment and the longest follow-up. The DCR is defined as the sum of CR+PR+SD. To ensure the accuracy and consistency of extracted data, a third reviewer (L, Y) double-checked the extracted data and was involved in resolving the disagreements.

Risk-of-bias assessment

For RCTs, we assessed the risk of bias through the revised Cochrane risk-of-bias tool for randomized trials (RoB2) tool [16], which evaluates five domains to determine the overall risk of bias for each study. For cohort and case-control studies, we used the Newcastle-Ottawa Scale (NOS) [17], assessing studies from three broad perspectives: election, comparability, and ascertainment.

Data synthesis

We conducted the meta-analysis using R version 4.4.2 (2024-10-31) [18]. We calculated weighted mean differences (WMDs) with 95% confidence intervals (CIs) for continuous outcomes and risk ratios (RRs) with 95% CIs for binary outcomes. Forest plots were provided to graphical overview of the data for outcomes. Cochran’s Q statistic was used to test for heterogeneity and the *I²* statistic quantified heterogeneity. A random-effects model was applied when heterogeneity was substantial (*I² *≥ 60%), and a fixed-effects model otherwise (*I²* < 60%). Subgroup analyses were conducted based on different types of pNETs and different types of PRRT, if sufficient data were available. If data were insufficient for meta-analysis, outcomes were analyzed descriptively.

Results

Search Results

We identified 8,096 records through electronic databases and 17 additional records from supplementary searches. After automatically removing 1,725 duplicates, we reviewed titles, abstracts, and full texts of the remaining 6,371 literature. Finally, nine studies met the criteria and were included in this review. The search process is shown in Figure 1.

**Figure 1:** Flow diagram of the search process. pNET, pancreatic neuroendocrine tumor; PRRT, peptide receptor radionuclide therapy

Study Characteristics and Risk-of-Bias Assessment

Of the nine included studies, only one (11.1%) was an RCT, and the remaining eight (88.9%) were cohort studies. The majority of studies were conducted in Italy (4, 44.4%), followed by the Netherlands (2, 22.2%), India (1, 11.1%), France (1, 11.1%), and a multi-center study in Europe (1, 11.1%). Regarding interventions/exposures and controls, four studies compared PRRT with other treatments, including surgery, SSAs, target agents (Sunitinib or Everolimus), and chemotherapy. Three studies compared different dosages of 177Lu-DOTATATE. One study compared 177Lu-DOTATATE plus capecitabine versus 177Lu-DOTATATE alone, and another compared salvage PRRT to only received initial PRRT. The median follow-up duration ranged from 25.7 to 88.6 months. Notably, three of the included studies were published as abstracts. The characteristics of the included studies are shown in Table 1.

**Table 1:** Characteristics of included studies. pNETs, pancreatic neuroendocrine tumors; PRRT, peptide receptor radionuclide therapy; G1-G2, WHO 2010 classification Grade 1 and Grade 2; SSAs, somatostatin analogs; CT, chemotherapy; I-PRRT, initial PRRT; R-PRRT, retreatment with PRRT; RR-PRRT, re-retreatment with PRRT

First author (year)	Country/region	Journal	Study design	Type of pNETs	Intervention/exposure	Control	No. of pNETs	Median follow-up duration	Risk-of-bias assessment
EANM’14 (2014) [19]	Italy	European Journal of Nuclear Medicine and Molecular Imaging	Prospective cohort (abstract)	Advanced G1-G2 pNETs	177Lu-DOTATATE reduced dosage	177Lu-DOTATATE full dosage	65	42 months	7
Ballal et al. (2017) [20]	India	Clinical Nuclear Medicine	Retrospective cohort	Advanced pNETs	177Lu-DOTATATE plus capecitabine	177Lu-DOTATATE only	49	32.4 months	7
Sansovini et al. (2017) [21]	Italy	European Journal of Nuclear Medicine and Molecular Imaging	Prospective cohort	Unresectable or metastatic G1-G2 pNETs	177Lu-DOTATATE full activity	177Lu-DOTATATE reduced activity	60	59 months	8
Lena et al. (2020) [22]	Italy	Endocrine Pathology	Retrospective cohort	Morphologically well-differentiated pNETs	PRRT (177Lu-DOTATATE and 90Y-DOTATOC)	Upfront surgery	48	PRRT group: 42 months; upfront surgery group: 69 months	7
Baudin et al. (2022) [23]	France	European Journal of Nuclear Medicine and Molecular Imaging	RCT (abstract)	Advanced pNETs	177Lu-Octreotate	Antiangiogenic agent (Sunitinib)	84	Not reported	High
Custodio et al. (2016) [24]	Europe	Neuroendocrinology	Retrospective cohort (abstract)	Advanced non-functional, well-differentiated pNETs	PRRT	SSAs^d^ or CT^e^ or target agents (Sunitinib or Everolimus)	210	Not reported	6
Genc et al. (2018) [25]	The Netherlands	World Journal of Surgery	Retrospective cohort	pNETs (without detailed definition)	PRRT	Surgery or CT or target agents or SSAs or no therapy	611	25.7 months	6
Sansovini et al. (2013) [26]	Italy	Neuroendocrinology	Prospective cohort	Advanced G1-G2 pNETs	177Lu-DOTATATE reduced dosage	177Lu-DOTATATE full dosage	52	Full-dosage group: 29 months; reduced dosage group: 26 months	8
van der Zwan et al. (2018) [27]	The Netherlands	European Journal of Nuclear Medicine and Molecular Imaging	Prospective cohort	Advanced pNETs	I-PRRT	R-PRRT or RR-PRRT or not undergoing salvage therapy	77	88.6 months	9

Among the eight cohort studies, the NOS scores ranged from 6 to 9 stars, with an average score of 7.25 stars. The only RCT study was assessed as high risk of bias.

Efficacy

PRRT Full Dosage vs. Reduced Dosage

The meta-analysis comparing full dosages versus reduced dosages of 177Lu-DOTATATE for G1-G2 pNETs revealed no significant differences between the two dosage regimens in terms of DCR (three studies, 177 patients, RR = 1.07, 95% CI 0.94-1.22), CR (three studies, 177 patients, RR = 3.23, 95% CI 0.91-11.54), PR (three studies, 177 patients, RR = 1.66, 95% CI 0.93-2.97), SD (three studies, 177 patients, RR = 0.79, 95% CI 0.60-1.04), and PD (two studies, 112 patients, RR = 0.66, 95% CI 0.30-1.47) between the full dosage and reduced dosage groups. Despite the lack of statistically significant differences, the full-dosage group showed superior efficacy compared to the reduced-dosage group (Figures 2-6).

**Figure 2:** Forest plots comparing full dosage (FD) vs. reduced dosage (RD) of PRRT for disease control rate. PRRT, peptide receptor radionuclide therapy; CI, confidence interval

**Figure 3:** Forest plots comparing full dosage (FD) vs. reduced dosage (RD) of PRRT for complete response. PRRT, peptide receptor radionuclide therapy; CI, confidence interval

**Figure 4:** Forest plots comparing full dosage (FD) vs. reduced dosage (RD) of PRRT for partial response. PRRT, peptide receptor radionuclide therapy; CI, confidence interval; RR, risk ratio

**Figure 5:** Forest plots comparing full dosage (FD) vs. reduced dosage (RD) of PRRT for stable disease. PRRT, peptide receptor radionuclide therapy; CI, confidence interval; RR, risk ratio

**Figure 6:** Forest plots comparing full dosage (FD) vs. reduced dosage (RD) of PRRT for progressive disease. PRRT, peptide receptor radionuclide therapy; CI, confidence interval; RR, risk ratio

Two of the three studies [19,21] reported PFS could not be pooled due to high levels of uncertainty or insufficient events, potentially leading to unreliable estimates. A study published in 2014 [19] indicated no significant difference in median PFS between the full dosage (46 months, 95% CI 26.0-69.0) and reduced dosage groups (25 months, 95% CI 20 to not reached) (*P *= 0.145). Similarly, a 2017 study [20] reported a median PFS of 53.4 months (95% CI 20.1-68.7) for the full-dosage group and 21.7 months (95% CI 18.1-48.2) (*P *= 0.353) for the reduced dosage group. Only one study [21] provided data on median OS, which showed a significant difference favoring the full-dosage group (not reached vs. 63.8 months, 95% CI 25.9 to not reached; *P *= 0.007).

PRRT vs. Other Treatments

The only included RCT, the OCLURANDOM phase II study [23], compared 177Lu-Octreotate (OCLU) and Sunitinib (SUN) in patients with advanced pNETs. The OCLU arm demonstrated a significant advantage, with a 12-month PFS rate of 80.5% (90% CI 67.5-89.9) compared to 42% (90% CI 29.1-55.5) in the SUN arm. The median PFS was also longer in the OCLU arm (20.7 months, 90% CI 17.2-23.7) compared to the SUN arm (11 months, 90% CI 8.8-12.4).

A retrospective cohort study [25] from the Netherlands Cancer Registry showed that pNETs who underwent surgery had the highest five-year survival rate (219/255, 86%) compared to those treated with PRRT (14/41, 33%), chemotherapy (9/44, 21%), targeted therapy (21, not reached), and SSAs (15/62, 24%), with all comparisons showing statistical significance (*P *< 0.001). Additionally, the median survival for patients receiving PRRT was the longest (43.6 months) compared to chemotherapy (7.6 months), target agents (16.2 months), SSAs (23.1 months), and surgery (36.2 months).

A multicenter European cohort [24] retrospectively analyzed advanced non-functional well-differentiated pNETs treated with various therapeutic strategies. The results showed that a longer PFS was observed in patients receiving PRRT (28.2 months; 95% CI 12.1-44.2) compared to those treated with SSAs (15.8 months; 95% CI 14.2-17.5), CT (12.1 months; 95% CI 8.6-15.6), or targeted agents (TA) (17.5 months; 95% CI 14.7-20.3) (*P* < 0.001).

PRRT vs. PRRT Plus Capecitabine

A retrospective cohort study [20] from India assessed the efficacy and safety of 177Lu-DOTATATE plus capecitabine (*n *= 23) versus 177Lu-DOTATATE alone (*n *= 26). The results showed that no patients achieved CR In both group; seven (30.4%) achieved PR in the combination therapy group, and two (7.7%) in the monotherapy group. SD was observed in 12 patients (52.2%) and 14 patients (53.8%), and PD was observed in two patients (8.7%) and eight patients (30.8%) in the 177Lu-DOTATATE plus capecitabine group and 177Lu-DOTATATE only group, respectively.

Salvage PRRT

A prospective cohort study from the Netherlands investigated the efficacy and safety of salvage treatment with 177Lu-DOTATATE [27]. Patients who initially received PRRT (I-PRRT) and later underwent salvage PRRT (R-PRRT) or re-treatment (RR-PRRT) upon disease progression were compared to those who only received I-PRRT. For pNETs receiving initial PRRT (I-PRRT), the median PFS was 32.7 months (95% CI 27.2-38.1), which showed no significant difference compared to the control group (39.1 months, 95%CI 31.8-46.5, *P *= 0.59). After receiving salvage PRRT, the median PFS for pNETs was 14.4 months (95% CI 11.5-17.2) for the R-PRRT group and 19.3 (95% CI 10.4-28.1) for the RR-PRRT group. Besides, the retreatment group showed a longer median OS compared to the control group. The combined median OS in patients receiving I-PRRT, R-PRRT, and RR-PRRT was 93.9 months (95% CI 39.4-148.3) vs 61.5 months (95% CI 49.9-73.2, *P *= 0.57).

Safety

Only a few studies reported safety outcomes. For full- versus reduced dosage of PRRT, no grades 3-4 hematological toxicity event (0/177) were reported in all three studies [19,21,26], and only one case of grades 3-4 renal toxicity (1/117) was observed in two studies [19,26].

In the OCLURANDOM trial [23], grade 3 or higher AEs were less frequent in the OCLU arm (18/41, 44%) compared to the SUN arm (26/43, 60%). The most common AEs included fatigue (3/41, 7%, vs. 5/43, 12%), reduced blood count (5/41, 12%, vs. 10/43, 24%), and hypertension (5/41, 12%, vs. 8/43, 19%).

Discussion 

This review systematically searched and assessed studies that compared the efficacy and safety of PRRT and other treatment protocols. Although the number of included studies was limited and the comparisons varied, our results suggest that PRRT demonstrates superior efficacy and safety compared to SSAs, chemotherapy, and target agents. Additionally, the full dosage of 177Lu-DOTATATE was found to be more effective and safer than the reduced dosage for G1-2 pNETs. As for patients with progressive disease, previously treated with PRRT, salvage PRRT also proved to be effective and safe.

Our meta-analysis indicates that PRRT, specifically 177Lu-DOTATATE, shows promising potential for treating advanced pNET patients, consistent with findings from other studies. A systematic review and meta-analysis [28] included 15 observational studies reported that 177Lu-DOTATATE achieved a higher DCR compared to Everolimus (81% vs. 73%, *P* < 0.01) and resulted in longer PFS (25.7 months vs. 14.7 months, *P* < 0.01). Pusceddu et al. retrospectively analyzed 508 patients with advanced, well-differentiated enteropancreatic NETs [29]. Their results showed that the median PFS was longer for patients receiving PRRT compared to those receiving chemotherapy or targeted therapy. For patients with pNETs specifically, the adjusted hazard ratio (aHR) was 0.41, indicating a 59% reduction in the risk of progression or death compared to chemotherapy or targeted therapy. Although there was a clinically meaningful improvement in OS for the PRRT group, no significant difference in OS was observed between the two treatment groups.

In Italian studies by Sansovini et al. provided data on patients receiving full dosage and reduced dosage of PRRT. The results reported that the full dosage of 27.8GBq brings to better PFS and should be considered the recommended dosage for advanced pNETs patients. Unlike this conclusion in pNETs, a 10-year follow-up study with 43 advanced G1-2 NETs patients [30] indicated that no significant difference in PFS was observed between patients receiving a reduced dose of 18.5 GBq and those receiving a full dose of 27.5 GBq, with both groups having a median PFS of 59.8 months. These findings highlight the need for further research to identify the optimal PRRT dosage in advanced pNETs and other types of NETs.

Salvage PRRT demonstrated efficacy and safety in patients with progressive pNETs, although no significant difference was found in OS, the retreatment group showed a longer median OS compared to the control group. This indicates that PRRT can serve not only as an initial treatment but also as a valuable option for subsequent therapy in cases of disease progression. Results from a systematic review and meta-analysis by Strosberg et al. further support the potential benefits of PRRT re-treatment in patients with progressive NETs [31]. Their findings indicate that the median PFS for patients undergoing re-treatment with 177Lu-PRRT was 12.52 months, with a DCR of 71%. Moreover, 177Lu-PRRT re-treatment demonstrated a safety profile comparable to that of initial PRRT. However, extra caution is required due to the potential for renal side effects associated with PRRT re-treatment. A retrospective cohort study by Emily et al. [32] analyzed 47 patients with NETs and showed that PRRT retreatment is generally safe and offers a valuable therapeutic option for patients with metastatic progressive NETs who have limited other treatment options. Nonetheless, the study reported that 17.2% of patients developed renal toxicity after PRRT2, including one patient who experienced grade 4 renal toxicity requiring dialysis. This highlights the need for careful monitoring of renal function in patients undergoing PRRT retreatment.

Limitations

This review also has several limitations. First, while we included eight observational cohort studies, we only identified one RCT (reported as an abstract) that met the inclusion criteria. The high risk of bias associated with this RCT, which is most likely attributable to the unpublished full text, limits the strength of conclusions that can be drawn from randomized evidence. Additionally, the heterogeneity in study designs and treatment protocols prevented us from conducting a meta-analysis for some outcomes, leaving us to rely on descriptive analysis instead. The review was restricted to studies published in English, which may have introduced language bias. Finally, we also included conference abstracts that contained data results. Since these studies were not published in peer-reviewed journals, their conclusions should be interpreted with caution. However, given the scarcity of comparative data in this field, these observational studies provide preliminary evidence to guide clinical decision-making. Future high-quality RCTs with larger sample sizes and standardized protocols are urgently needed to validate these findings.

Implications

The findings of this review have some implications for clinical practice. PRRT should be considered a valuable treatment option for patients with advanced pNETs, particularly for those who are not candidates for surgery or have failed other therapies. The evidence supports the use of 177Lu-DOTATATE as an effective agent for prolonging PFS and OS, with a favorable safety profile. While reduced doses of PRRT also showed activity, full dosage may bring better efficacy and safety for patients with advanced G1-2 pNETs.

For researchers in this field, we recommend that future studies focus on the following areas: (1) the potential benefits of combination therapies involving PRRT; (2) the efficacy of PRRT across different types of pNET patients; and (3) the comparative efficacy of various PRRT agents. High-quality RCTs with larger sample sizes and prolonged follow-up periods are essential to confirm these results and further explore the optimal use of PRRT in treating advanced pNETs.

## Conclusions

This systematic review and meta-analysis synthesizes evidence supporting PRRT as a clinically valuable treatment for advanced pNETs, demonstrating favorable efficacy and safety compared to conventional therapies based on the low quality of evidence. Our findings indicate that PRRT, particularly 177Lu-DOTATATE, is associated with prolonged PFS and OS relative to chemotherapy, targeted agents, and somatostatin analogs. Notably, full-dose PRRT regimens showed superior efficacy in tumor control (e.g., higher disease control rates and longer median OS) compared to reduced doses, with no significant increase in severe hematological or renal toxicity, reinforcing its role as a balanced therapeutic option. Additionally, salvage PRRT and combination therapies (e.g., PRRT with capecitabine) exhibited promising activity in progressive or refractory cases, further expanding its clinical utility. However, the conclusions are constrained by the predominance of observational studies (8/9) and the inclusion of only one RCT with a high risk of bias. Heterogeneity in treatment protocols and the reliance on retrospective data limit the generalizability of these findings. Future research should prioritize large-scale RCTs to validate optimal dosing strategies, compare PRRT with emerging therapies, and evaluate long-term safety profiles, particularly regarding renal function in retreatment settings. Despite these limitations, our analysis underscores PRRT as a pivotal option for inoperable or advanced pNETs, advocating for its integration into personalized treatment algorithms while awaiting confirmatory evidence.

## Appendices

Appendix: Search strategy (searched up to June 12, 2024)

**Table 2:** Search strategy (searched up to 12th Jun 2024)

PubMed
#1. "Peptide Receptor Radionuclide Therapy"[Title/Abstract]
#2. "PRRT"[Title/Abstract]
#3. "DOTATOC"[Title/Abstract]
#4. "DOTATATE"[Title/Abstract])
#5. OR/#1-#4
#6. "pancreatic neuroendocrine tumor*"[Title/Abstract]
#7. "pancreatic neuroendocrine neoplasm*"[Title/Abstract]
#8. "pannet*"[Title/Abstract]
#9. "pnet*"[Title/Abstract]
#10."Pancreatic Neoplasms"[MeSH Terms]
#11."Neuroendocrine Tumors"[MeSH Terms]
#12.OR/#6-#11
#13.#5 AND #12
Embase
#1. 'pancreas tumor'/exp
#2. 'neuroendocrine tumor'/exp
#3. 'pancreatic neuroendocrine tumor*':ab,kw,ti
#4. 'pancreatic neuroendocrine neoplasm*':ab,kw,ti
#5. 'pannet*':ab,kw,ti
#6. 'pnet*':ab,kw,ti
#7. OR/#1-#6
#8. 'peptide receptor radionuclide therapy'/exp
#9. 'dotatate':ab,kw,ti
#10.'dotatoc':ab,kw,ti
#11.'prrt':ab,kw,ti
#12.OR/#8-#11
#13.#7 AND #12
Cochrane
#1. MeSH descriptor: [Pancreatic Neoplasms] explode all trees
#2. MeSH descriptor: [Neuroendocrine Tumors] explode all trees
#3. ('pancreatic neuroendocrine tumor'):ti,ab,kw (Word variations have been searched)
#4. ('pancreatic neuroendocrine neoplasm'):ti,ab,kw (Word variations have been searched)
#5. ('pannet'):ti,ab,kw (Word variations have been searched)
#6. ('pnet'):ti,ab,kw (Word variations have been searched)
#7. OR/#1-#6
#8. ('Peptide Receptor Radionuclide Therapy'):ti,ab,kw (Word variations have been searched)
#9. ('prrt'):ti,ab,kw (Word variations have been searched)
#10.('DOTATOC'):ti,ab,kw (Word variations have been searched)
#11.('DOTATATE'):ti,ab,kw (Word variations have been searched)
#12.OR/#8-#12
#13.#7 AND #12
Web of Science
#1. TS=('Peptide Receptor Radionuclide Therapy')
#2. TS=('prrt')
#3. TS=('DOTATOC')
#4. TS=('DOTATATE')
#5. OR/#1-#4
#6. TS=('pancreatic neuroendocrine tumor*')
#7. TS=('pancreatic neuroendocrine neoplasm')
#8. TS=('pannet*')
#9. TS=('pnet*')
#10.OR/#6-#9
#11.#5 AND #10
